The article "Enteral Nutrition: Based on the Combination of Nutrison Fibre and TPF-DM with A Marine Biological-Based Active Polysaccharide Preparation" was published in 2022. Journal: Comput Math Methods Med.

# Enteral Nutrition: Based on the Combination of Nutrison Fibre and TPF-DM with A Marine Biological-Based Active Polysaccharide Preparation

**DOI:** 10.1155/2022/6213716

**Published:** 2022-06-30

**Authors:** Qiuyue Tang, Yaqin Cheng

**Affiliations:** Department of Neurology, Affiliated Hospital of Nantong University, Nantong, Jiangsu 226000, China

## Abstract

Good nutrition is essential for human growth, wound healing, and spiritual vitality. However, some individuals are unable to eat or experience gastrointestinal problems such as severe diarrhea, vomiting, gastric retention, and even gastrointestinal bleeding for a variety of causes. Therefore, it has important clinical significance to provide patients with required nutrients and maintain the integrity of the body's tissues and organs through enteral nutrition. Based on this, this work uses a dual carrier of polylactic acid (PLA) and polyvinyl alcohol (PVA) to carry marine biopolysaccharides combined with sodium alginate (PSS) and successfully obtains the intestinal tract based on marine bioactive polysaccharides. Nutritional oral biological preparations (PSS-PLA/PVA) also cooperate with enteral nutritional suspension (diabetes) (TPF-DM) and Nutrison fibre to provide enteral nutritional support for critically ill patients. PSS-PLA/PVA has been shown in clinical studies to increase the effect of enteral nutrition support, the function of intestinal T lymphatic tissue, and the ability to control immunological function, indicating that it is worthy of further clinical development.

## 1. Introduction

As a disease with high mortality and disability rate among middle-aged and elderly people, the incidence rate of neurocritical disease, with the development of population aging, is gradually increasing. The main clinical features are impaired cognitive function, central fever, dysphagia, and limb dysfunction. In addition, neurocritical illness is prone to induce severe stress reactions, accelerates the body's metabolic decomposition, and causes complications such as malnutrition and hypoproteinemia in patients, which are the primary factors restricting the prognosis and survival rate of patients. Compared with other diseases, critically ill patients are susceptible to the effects of drugs and stress reactions, leading to impaired gastrointestinal function, leading to diarrhea, vomiting, gastric retention, and even gastrointestinal bleeding [1, 2]. Therefore, nutritional support is necessary to regulate the immune function of the patient's body and maintain the functional integrity of the body's tissues and organs [3–6].

Nutritional support can be divided into two types, enteral and parenteral [7]. Vitamins, calories, electrolytes, amino acids, and trace elements are delivered to patients via intravenous channels through parenteral nutrition [8–11]. However, using parenteral nutrition exclusively will make it more difficult to maintain patients' nutritional status and raise the risk of problems [12–15]. Enteral nutrition (EN) is a way to provide patients with required nutrients through the gastrointestinal route [16, 17]. In the early stages of neurocritical patients, enteral nutrition can better maintain the integrity of the body's tissues and organs than parenteral nutrition and has a nonnegligible impact on the prognosis of patients [18]. In addition, enteral nutrition in the early stage of the patient can effectively increase the blood flow of the gastric mucosa and maintain the barrier function of the gastrointestinal mucosa. At the same time, food entering the gastrointestinal tract can also stimulate the body's advocacy-neuro-endocrine immune axis, effectively preventing the liver cholestasis situation. In addition, enteral nutrition can slow down the body's stress response, maintain the function of the intestinal mucosa, and reduce the occurrence of side effects such as gastrointestinal bleeding [19]. Enteral nutritional suspension (diabetes) (TPF-DM) and Nutrison fibre are commonly used clinical enteral nutrition drugs. In addition to supplying energy to the body, they can also control the patient's blood sugar and blood lipids and have a better therapeutic effect on critically ill patients. However, the use of TPF-DM and Nutrison fibre alone can easily produce side effects such as abdominal distension, diarrhea, and malabsorption. Therefore, how to improve this phenomenon is a hot issue of current research.

According to various sources, marine biological polysaccharides can be classified as marine plant polysaccharides, marine animal polysaccharides, and marine microbial polysaccharides [20–22]. The most researched marine polysaccharides include algae polysaccharides, scallop glycosaminoglycans, mussel polysaccharides, abalone polysaccharides, and YCP polysaccharides extracted from the mycelium of marine fungus Ys4108. Because of its unique chemical composition and structure, marine biopolysaccharides usually have antioxidant, antithrombotic, immune regulation, cholesterol-lowering, and antitumor effects [23–25]. It possesses dietary fibre qualities, and as an EN preparation, it can aid in the absorption of carbs, lipids, vitamins, and minerals by the body. At the same time, by increasing the activity of immune cells, marine polysaccharides can increase the secretion of cytokines, causing the body to manufacture antibodies to improve immunological function. In addition, the dietary fibre components contained in marine biopolysaccharides can effectively control the increase in blood sugar and improve glucose tolerance and cholesterol content. Therefore, in this work, sodium alginate (PSS) was selected as the main component of marine biobased active polysaccharide enteral nutrition preparation, and polylactic acid (PLA) and polyvinyl alcohol (PVA) were used as drug carriers to prepare a new type of marine organism. Active polysaccharide oral preparation was used in combination with TPF-DM and Nutrison fibre, in order to improve the side effects of TPF-DM and Nutrison fibre as enteral nutrition preparations and to investigate its application effect in neurocritical patients.

The paper is organized as follows: the materials and methods are presented in Section 2.  Section 3 discusses the experimental analysis and results of the proposed concepts. Finally, in Section 4, the research work is concluded.

## 2. Materials and Methods

In this section, we define the reagents, instruments, preparation of PSS-PLA/PVA, analysis of PSS-PLA/PVA drug release ability *in vitro*, clinical research, and statistical analysis in detail.

### 2.1. Reagents

PSS was purchased from Shanghai Fusheng Industrial Co., Ltd. (Shanghai, China). PLA and PVA are provided by Wuhan Haishan Technology Co., Ltd. (Hubei, China). Dichloromethane, hydrochloric acid, potassium dihydrogen phosphate, and sodium hydroxide were purchased from Jinan Chuangshi Chemical Co., Ltd. (Shandong, China). Trypsin and pepsin were produced by Wuhan Zeshancheng Biomedical Technology Co., Ltd. (Hubei, China). TPF-DM and Nutrison fibre were provided by Nutricia Pharmaceutical (Wuxi) Co., Ltd. (Jiangsu, China).

### 2.2. Instrument

The KQ-500E ultrasonic cleaner was purchased from Kunshan Ultrasonic Instrument Co., Ltd. (Jiangsu, China). The micro high-speed refrigerated centrifuge C1650R-230V was provided by Lepto Scientific Instruments (Beijing) Co., Ltd. (Beijing, China). Carl Zeiss provided the SIGMA 500 field emission scanning electron microscope (Oberkochen, Germany). Particle Sizing Systems sold the AccuSizer780 AD multipurpose automatic counting particle size detector (Florida, USA). An Oulaibo constant temperature oscillator OLB-100B was purchased from Jinan Oulaibo Scientific Instrument Co., Ltd. (Shandong, Jinan).

### 2.3. Preparation of PSS-PLA/PVA

PSS-PLA is prepared by a double emulsification solvent evaporation method. 50 mg of PSS was dissolved in 1.0 mL of double-distilled water to prepare the PSS solution. Prepare a PLA solution with a concentration of 40 mg/mL using dichloromethane as the solvent. And use double-distilled water to prepare 4.0 mg/mL and 1.0 mg/mL PVA solutions. The PSS solution was progressively dripped into the PLA solution under ultrasonography in an ice bath to obtain a uniformly dispersed emulsion. Under the same conditions, it was slowly added to the 4.0 mg/mL PVA solution and added to 1.0 mg/mL PVA solution under the condition of stirring in the ice bath. Stir overnight, then freeze centrifugation at 12,000 rpm for 20 min, discard the supernatant, wash the precipitate with double-distilled water, and freeze-dry to obtain the PSS-PLA/PVA oral preparation. And use the field emission scanning electron microscope SIGMA 500 to characterize it.

### 2.4. Analysis of PSS-PLA/PVA Drug Release Ability *In Vitro*

The artificial gastric juice is prepared by adding 8.2 mL of dilute hydrochloric acid and 5.0 g of pepsin to 400 mL of double-distilled water. After stirring, add double-distilled water and dilute to 500 mL. The artificial intestinal juice is prepared by dissolving 3.9 g of potassium dihydrogen phosphate in 250 mL of double-distilled water, using 0.1 mol/L sodium hydroxide to adjust the pH = 6.8, and dissolving another 5.0 g of trypsin in double-distilled water. After mixing the two solutions, dilute to 500 mL with double-distilled water to obtain artificial intestinal juice. Place the PSS-PLA/PVA preparation in 10 mL of artificial gastric juice or artificial intestinal juice, and oscillate at a speed of 150 rpm in a constant temperature shaker at 37°C. Take out 1.0 mL of artificial intestinal juice or gastric juice at 120, 240, 480, and 720 min, and centrifuge at 12,000 rpm. Take the supernatant to detect its absorbance at 490 nm, and calculate the PSS-PLA/PVA preparation in the artificial gastric juice and cumulative release rate in intestinal juice.

### 2.5. Clinical Research

In this section, we define the general data analysis, treatment method, and observation index in detail.

#### 2.5.1. General Data Analysis

A total of 323 neurocritical patients who were treated in our hospital from December 2019 to February 2021 were selected, including 219 male patients and 104 female patients, with an average age of 63.4 ± 14.6 years. The specific patient information is recorded in Table 1.

Before the patients receive enteral nutrition support, use the Acute Physiology and Chronic Health Score II (APACHE II) to make a comprehensive assessment of their vital signs, oxygenation, whether there is chronic organ dysfunction, whether they are in a state of immunosuppression, etc., where APACHE II score ≥ 16 points can be included in the observation. In addition, patients with severe heart disease, digestive system disease, endocrine disease, liver and kidney dysfunction, and unstable vascular dynamics besides neurocritical disease were not included in the observation. Relevant clinical treatments in this study have been approved by the hospital ethics committee, and all patients and their families have signed an informed consent form.

#### 2.5.2. Treatment Method

All patients were divided into four groups according to the nutritional risk screening score before enteral nutrition support (NRS2002) and different nutritional support methods, and the total calories of enteral nutrition was 25 kcal/(kg·d), with continuous treatment for 7 days. Among them, the group with the NRS2002 score < 3 points and two enteral nutrition suspensions (TPF-DM and Nutrison fibre) is low-risk group 1, and two enteral nutrition suspensions plus PSS-PLA/PVA oral preparations are used. The second group is the low-risk group; the group with NRS2002 score ≥ 3 and two enteral nutrition suspensions is high-risk group 1, and the group is treated with two enteral nutrition suspensions plus PSS-PLA/PVA oral preparations. Its treatment mechanism for patients is shown in Figure 1.

#### 2.5.3. Observation Index

Before and after the nutritional support was given, the patient's albumin (ALB), prealbumin (pre-ALB), and hemoglobin (HB) were tested for biochemical indicators used to evaluate the patient's nutritional support. Also, the total number of T lymphocytes (TLC) levels is used to evaluate the effect of enteral nutrition on lymphocyte function, and the levels of IgA, IgG, and IgM are used to evaluate the effect of enteral nutrition on the immune function of critically ill patients. Furthermore, gastrointestinal symptoms such as gastrointestinal haemorrhage, diarrhea, constipation, lung infection, vomiting, and stomach retention were recorded.

### 2.6. Statistical Analysis

Use SPSS 22.0 to process and analyze the data involved in this research. Quantitative variables are expressed as mean ± standard deviation, and qualitative variables are described by frequency distribution and percentage (%). The *t*-test is used for the analysis of quantitative variables, and the analysis of qualitative variables uses the *χ*^2^ test. *P* < 0.05 indicates statistical significance.

## 3. Results and Discussion

### 3.1. PSS-PLA/PVA Morphology Characteristics

The morphology of the marine biobased active polysaccharide preparation—PSS-PLA/PVA preparation—was characterized by scanning electron microscopy.  Figure 2 shows that the whole of PSS-PLA/PVA is spherical and evenly dispersed. The particle size distribution results show that the average particle size of PSS-PLA/PVA is 173.52 ± 23.69 nm, and the average potential is −19.63 ± 3.62 mV. Its small particle size can be effectively absorbed by the body and improve the effect of enteral nutrition.

### 3.2. *In Vitro* Release Effect of PSS-PLA/PVA

In order to simulate the release of PSS-PLA/PVA in the body, the cumulative release rate of PSS-PLA/PVA in artificial gastric juice and artificial intestinal juice was investigated, respectively (Figure 3). The results show that the drug release rate of PSS-PLA/PVA is faster at 0−60 min and then tends to be flat, and the cumulative release of PSS-PLA/PVA in artificial gastric juice at 720 min is only 26.31%, while at 720 min, the cumulative release amount in artificial intestinal fluid was 69.62%. This result proves that compared with gastric juice, PSS-PLA/PVA is easier to release in the intestine and can meet its enteral nutrition standard.

### 3.3. Evaluation of the Effect of Enteral Nutrition

In order to evaluate the effects of PSS-PLA/PVA oral preparations on enteral nutrition, ALB, HB, and pre-ALB were used as nutritional evaluation indicators to investigate their therapeutic effects on patients with different risk levels (Figure 4). The treatment results showed that each group of drugs had a significant therapeutic effect on neurocritical patients (*P* < 0.05). In addition, the same drug has different effects on the low-risk group and the high-risk group, and it has a better therapeutic effect on patients in the high-risk group. In addition, compared with only using TPF-DM and Nutrison fibre, the addition of PSS-PLA/PVA oral preparations can improve the patient's enteral nutrition absorption.

### 3.4. T Lymphocyte Function Evaluation

TLC is employed as an evaluation index to evaluate the impact of different medicines on the T lymphatic function of neurocritical patients with varied risks, because enteral nutrition can sustain the function of the intestinal lymphatic tissue of patients (Figure 5). The results showed that compared with before treatment, the number of TLC in neurocritical patients with different risk levels increased after different drug treatments (*P* < 0.05). And compared with only using TPF-DM and Nutrison fibre, the combination of TPF-DM and Nutrison fibre with PSS-PLA/PVA oral preparation has better therapeutic effect.

### 3.5. Patient's Immune Function Regulation

IgA, IgG, and IgM are all types of immunoglobulins. Therefore, this study used the levels of IgA, IgG, and IgM in neurocritically ill patients as indicators to investigate the effect of enteral nutrition on the immune function of patients (Figure 6). The findings revealed that after therapy, the immunoglobulin levels of patients in each group increased (*P* < 0.05), with the increase being more pronounced in the high-risk group. In addition, the addition of PSS-PLA/PVA oral preparations can improve the regulatory effect of TPF-DM and Nutrison fibre on immune function.

### 3.6. Incidence of Gastrointestinal Reactions in Patients

As neurocritical patients are prone to adverse reactions such as diarrhea, constipation, vomiting, lung infection, gastrointestinal bleeding, gastric retention, and even death after treatment, the influence of enteral nutrition on the incidence of adverse reactions was investigated (Figure 7). The results show that the addition of PSS-PLA/PVA oral preparations can reduce the occurrence of adverse reactions.

### 3.7. Discussion

In the care of critically ill patients, malnutrition usually leads to reduced efficacy of drug treatment and some side effects. Therefore, strengthening the nutritional support for critically ill patients is essential. Studies have found that enteral nutrition can effectively improve the metabolic abnormalities of critically ill patients and reduce the risk of complications during treatment [26], especially in patients with neurological diseases such as stroke and dementia and patients who require mechanical ventilation [27–29]. Enteral nutrition can be divided into two types: oral and via catheter. Oral administration is typically utilised for patients who are able to swallow on their own, whereas transcatheter infusion is separated into a nasogastric tube and oral feeding tube. Patients who require short-term enteral nutrition support should use a nasogastric tube, whereas patients who require long-term enteral nutrition support should use an oral feeding tube. It is suitable for patients who have undergone partial or complete gastrectomy and who are at risk of aspiration.

In this work, two types of enteral nutrition were used to provide nutritional support to patients undergoing neurocritical treatment. One of the enteral nutrition support methods is the combined use of TPF-DM and Nutrison fibre, and the other enteral nutrition support method is the use of Nutrison fibre and TPF-DM in combination with a marine biobased active polysaccharide preparation-PSS-PLA/PVA oral preparation. According to the NRS2002 score, patients were divided into low-risk and high-risk groups. Nutrition evaluation indicators such as ALB, pre-ALB, HB, TLC levels, and IgA, IgA, and IgA used to evaluate the regulatory effects of enteral nutrition on the immune function of critically ill patients were used. The detection results of IgG and IgM levels can find that each group of drugs has a significant therapeutic effect on neurocritical patients (*P* < 0.05). And the same drugs are more effective in treating patients in the high-risk group. Furthermore, when compared to only using TPF-DM and Nutrison fibre, adding PSS-PLA/PVA oral preparations can improve the patient's enteral nutrition support effect, maintain the function of intestinal T lymphatic tissue, and regulate the immune function of critically ill patients. In addition, the addition of PSS-PLA/PVA oral preparations can also effectively reduce the incidence of gastrointestinal reactions such as gastrointestinal bleeding, diarrhea, constipation, lung infection, vomiting, and gastric retention. This discovery provides a new way of enteral nutrition support for clinically critically ill patients.

## 4. Conclusion

PSS was used as the principal component of a marine bioactive polysaccharide enteral nutrition preparation in this work, with PLA and PVA serving as drug transporters to create a new form of marine bioactive polysaccharide oral preparation. The results show that compared with the combined effect of TPF-DM and Nutrison fibre, the addition of PSS-PLA/PVA has better enteral nutrition support effect for patients with different risk levels of neurocritical patients, maintaining the function of intestinal T lymphatic tissue and regulating the immune function of neurocritical patients. It is worthy of further clinical promotion and use.

## Figures and Tables

**Figure 1:** Enteral nutrition administration and absorption route.

**Figure 2:** Characterization of a novel oral preparation of marine biologically active polysaccharide-sodium alginate-polylactic acid/polyvinyl alcohol (PSS-PLA/PVA): (a) electron microscopy characterization diagram; (b) graph of particle size distribution.

**Figure 3:** Analysis of the cumulative release rate of polysaccharide-sodium alginate-polylactic acid/polyvinyl alcohol (PSS-PLA/PVA) in artificial gastric juice and artificial intestinal juice.

**Figure 4:** The effect of enteral nutrition on nutritional evaluation indexes of patients with different degrees of risk: (a) the effect on albumin (ALB) content; (b) the effect on hemoglobin (HB) content; (c) the effect on prealbumin (pre-ALB) content. ^∗^*P* < 0.05.

**Figure 5:** The effect of enteral nutrition on the total number of T cells (TLC) in patients with different degrees of risk.

**Figure 6:** The effect of enteral nutrition on the immune function of patients with different degrees of risk: (a) the effect on immunoglobulin A content; (b) the effect on immunoglobulin G content; (c) the effect on immunoglobulin M content.

**Figure 7:** The effect of enteral nutrition on the incidence of gastrointestinal reactions in patients.

**Table 1:** General data analysis.

	Group			
	Low risk 1 (*n* = 94)	Low risk 2 (*n* = 85)	High risk 1 (*n* = 77)	High risk 2 (*n* = 77)
Sex				
Male	58	61	52	48
Female	26	24	25	29
Age (years)	55.44 ± 11.52	57.63 ± 10.69	72.17 ± 11.68	71.56 ± 11.68
NRS2002 score	2	2	3.25 ± 0.62	3.56 ± 0.73
NIHSS score	8.89 ± 5.30	8.67 ± 4.28	13.56 ± 10.74	13.68 ± 9.84
GCS score	11.64 ± 3.44	12.65 ± 3.39	10.36 ± 4.37	10.68 ± 4.59

## Data Availability

The dataset used in this paper are available from the corresponding author upon request.
